The article "The Effects of Combuxil and Leizumab on Retinal Function and Serum Interleukin-17A in Premature Infants with Retinopathy" was published in 2022. Journal: Comput Math Methods Med.

# The Effects of Combuxil and Leizumab on Retinal Function and Serum Interleukin-17A in Premature Infants with Retinopathy

**DOI:** 10.1155/2022/6371994

**Published:** 2022-09-26

**Authors:** Huixuan Ren, Gang Su, Shunian Xu, Li Zhou, Shanjun Cai

**Affiliations:** ^1^Ophthalmology, Department of Ophthalmology, Affiliated Hospital of Zunyi Medical University, Guizhou Provincial Eye Hospital, Guizhou Branch Center of National Clinical Research Center for Eye Diseases, Guizhou Provincial Key Laboratory of Characteristic Eye Diseases Characteristics, Zunyi, Guizhou 563003, China; ^2^Ophthalmology, Affiliated Hospital of Zunyi Medical University, Zunyi, Guizhou 563003, China

## Abstract

**Objective:**

To investigate the effects of Compaximab and raizumab on retinal function and serum interleukin-17A level in retinopathy of prematurity.

**Methods:**

Sixty cases of retinopathy of prematurity treated in our hospital from February 2019 to April 2021 were selected. The patients were randomly divided into control group (*n* = 30) and research group (*n* = 30). The control group was treated with Compaq and the research group was treated with razumab. The curative effect, retinal function, incidence of complications, intraocular pressure at different time, and the level of serum interleukin-17A were compared.

**Results:**

Compared with the two groups, the curative effect of the research group 93.33% (28/30) was greater than that of the control group 66.67% (20/30), and the difference was statistically significant (*P* < 0.05). Compared with the incidence of complications, the incidence of corneal opacity, lens opacity, preretinal and vitreous hemorrhage, endophthalmitis, and traction retinal detachment in the research group was greatly lower, and the difference was statistically significant (*P* < 0.05). Following the therapy, the IOP of the two groups decreased at different times. The IOP of 1 min, 10 min, and 30 min in the research group was obviously lower, and the difference was statistically significant (*P* < 0.05). Following treatments, the levels of serum IL-17A were decreased. Compared with the control group, the level of serum IL-17A in the research group was greatly downregulated, and the difference was statistically significant (*P* < 0.05).

**Conclusion:**

Intravitreal injection of razumab is an effective treatment for retinopathy of prematurity, which can effectively improve the retinal function of infants. The level of serum interleukin-17A can be reduced and intraocular pressure can be regulated, which is safe and effective.

## 1. Introduction

Retinopathy of prematurity (ROP), formerly known as posterior lens fibroplasia, was first proposed by Terry. It is characterized by abnormal growth of retinal vessels at the junction of vascularized and nonvascularized areas of the retina [1, 2]. According to a retrospective analysis of the causes of visual impairment in children abroad, the blindness rate caused by ROP is as high as 8%. The rate of blindness can be reduced through early detection and timely treatment of ROP. The rate of blindness is high, so it has attracted more and more attention of pediatricians all over the world. Globally, there were about 184700 new ROP patients in 2010. About 20000 patients became blind or developed severe visual impairment as a result of ROP, and 12300 developed mild to moderate visual impairment [3]. ROP is a blindness disease. The main cause of blindness is retinal detachment caused by retinal vascular abnormality and scar formation. At present, hyperoxia exposure, small gestational age and low birth weight have been confirmed to be the main risk factors for retinopathy of prematurity [4, 5].

The article "The Effects of Combuxil and Leizumab on Retinal Function and Serum Interleukin-17A in Premature Infants with Retinopathy" was published in 2022. Journal: Comput Math Methods Med.

The main pathological changes of ROP are the arrest of normal retinal vascular development and pathological neovascularization, which can lead to blindness of retinal detachment in severe cases. In addition, the duration of mechanical ventilation, blood transfusion, use of caffeine, and serious complications such as respiratory distress syndrome (NRDS), bronchopulmonary dysplasia (BPD), maternal pregnancy induced hypertension, and prenatal hormone use were also confirmed to be related to the occurrence of ROP [6]. The pathogenesis of ROP is still unclear. It is generally believed that postnatal hyperoxia exposure on the one hand stops the development of normal retinal vessels. On the other hand, with the development of the disease, hypoxia causes excessive production of angiogenic factors in the body, which leads to pathological angiogenesis. It is suggested that inflammatory factors play an important role in blocking normal retinal vascular development, inducing pathological neovascularization, and promoting the occurrence of ROP. Some studies have shown that the levels of endothelial nitric oxide synthase, dicarboxylic acid carnitine (C3DC), glycine, and serine are significantly increased in children with ROP. Other biomarkers such as brain-derived neurotrophic factor and matrix metalloproteinase-9 (MMP-9) are still being studied. At present, a few foreign studies have confirmed that IL-17A is related to ocular neovascularization [7] and IL-17-related cytokines have also been confirmed to be involved in the pathological process of ROP [8], but its underlying mechanism is still unclear.

Previous studies at home and abroad have found that VEGF has been well explained in many animal models and humans [9–11]. Both razumab and bevacizumab are humanized monoclonal VEGF antibody fragments against retinal vascular diseases. Comperxil is a recombinant fusion protein with fully humanized amino acid sequence, which has become another choice for ROP therapy. Combuxil showed higher VEGF binding ability because it binds to the second Ig domain of VEGF receptor-1 [12]. Prospective study follow-up for 1 year found good anatomical structure and functional outcome of retina can be obtained after Compaq treatment of ROP [13]. Previously, some scholars have conducted a small sample study on the treatment of ROP by intravitreal injection of Combuxil. The results show that Compaq has less effect on intraocular pressure, but the efficacy and safety of larger samples after treatment, especially the effect on growth and development after treatment with Combuxil is still unclear [14]. The common dose of anti-VEGF of ROP is half that of adults, but VEGF is very important for neonatal development, especially for the development of brain, kidney, lung, and other important organs. The half-life of Compaximab is longer and its molecular weight is larger than that of razumab, which may have a greater negative effect on the growth and development of premature infants [15]. Therefore, Compaximab and raizumab were used to treat ROP, and the efficacy, safety, growth, and development parameters were evaluated and compared in order to delivery effective references for the follow-up of ROP. This study was to investigate the effects of Compaximab and raizumab on retinal function and serum interleukin-17A level in retinopathy of prematurity.

The article "The Effects of Combuxil and Leizumab on Retinal Function and Serum Interleukin-17A in Premature Infants with Retinopathy" was published in 2022. Journal: Comput Math Methods Med.

## 2. Materials and Methods

### 2.1. General Information

Sixty cases of retinopathy of prematurity from February 2019 to June 2021 were enrolled. The control group (*n* = 30) were treated with Compaq, and the study participants were treated with razumab. The controlled gestational age was 25-33 weeks, including 18 males and 12 females. In the research group (*n* = 30), the gestational age was 25-33 weeks, including 16 males and 14 females. This study was approved by the ethics committee of the hospital. All the guardians of the participants consent with the study.

Selection criteria: (1) according to the 2014 Chinese guidelines for screening retinopathy of prematurity [16], after the diagnosis of threshold lesion or type 1 prethreshold lesion, treatment should be received within 72 hours as far as possible. Threshold disease: Stage 3 + in area I or II and the adjacent lesions lasted for at least 5 hours or accumulate up to 8 hours, it was a disease that must be treated. Prethreshold disease: referred to the severity of ROP lesions that were obvious but have not reached the threshold, it can be divided into “type 1 pre-threshold lesion” and “type 2 pre-threshold lesion”. Type 1 prethreshold lesions included any stage lesions in area I with additional lesions, stage 3. Aggressive posterior ROP (AP-ROP): it occurs in the posterior pole, usually in area I, with rapid progress and often involving four quadrants. The disease may not progress according to the typical development law of stage 1 to 3, and the severe “additional lesion” was once called “Rush” disease; it often occurred in very low-weight premature infants. The condition was often more serious and needs to be treated as soon as possible. (2) Good compliance and can cooperate with the examiner during the follow-up period.

The article "The Effects of Combuxil and Leizumab on Retinal Function and Serum Interleukin-17A in Premature Infants with Retinopathy" was published in 2022. Journal: Comput Math Methods Med.

Exclusion criteria: (1) premature infants with ROP4 and stage 5 retinal detachment, and other retinal choroidopathy, those with congenital cataract or corneal leukoplakia and other serious ocular diseases, could not observe the fundus condition, and those with severe systemic diseases had no history of other eye surgery and external injuries. (2) Uncooperative treatment and lost patients during follow-up. (3) It did not meet the treatment standard of China's guidelines for screening retinopathy of prematurity.

### 2.2. Methods

All the children were treated with vitreous injection under surface anesthesia in the aseptic laminar flow operating room of our hospital. The infants were fasted for 2 hours before operation, and compound tropicamide eye drop was used for 3 times (10 min/times). After 3 times (5 min/times) of surface anesthesia with promevacaine hydrochloride eye drops, 5% povidone iodine solution was used to disinfect the eyes. The eyelid was opened with special eyelid opener for children, and the eyeball was fixed with ophthalmic micro tweezers. The 30G injection needle was injected into the 1 mm parallel optic axis behind the temporal limbus of the eyes. The control cases were injected by Compaq 0.25 mg. The research group received injection of 0.25 mg tobramycin dexamethasone eye ointment. Three days after operation, routine antibiotic eye drops were used.

### 2.3. Observation Indicators

#### 2.3.1. Curative Effect

The curative effect was judged by observing the anatomical outcome [17]. Effective: retrogression of additional lesions, tortuosity of retinal vessels, disappearance or decrease of neovascularization, and growth of normal retinal vessels around; ineffective: during the follow-up period, the recurrence of the disease requires reinjection or laser treatment, abnormal lesions such as crest and additional lesions relapse. Total effective rate = number of valid cases/total number of cases × 100%.

The article "The Effects of Combuxil and Leizumab on Retinal Function and Serum Interleukin-17A in Premature Infants with Retinopathy" was published in 2022. Journal: Comput Math Methods Med.

#### 2.3.2. Incidence of Adverse Reactions

The adverse reactions were compared during treatment, including ocular complications, corneal haze implantation, lens opacity, preretinal and intravitreous hemorrhage, endophthalmitis, and traction retinal detachment.

#### 2.3.3. Intraocular Pressure at Different Time

Intraocular pressure (IOP) was measured and recorded with Icare magnetic rebound tonometer (Icare, Finland) 1 minute before treatment and 1, 10, and 30 minutes after treatment.

#### 2.3.4. Serum IL-17A Level

Venous blood 1 ml was collected before treatment, on the 1st day and 15th day after treatment. The content of IL-17A in serum was determined by ELISA (ebioscience, USA). The content was determined according to the instructions of the kit.

### 2.4. Statistical Analysis

IBMSPSS24.0 software was applied for statistical analysis. The measurement data were expressed by mean ± standard deviation. The counting data were expressed by frequency or rate. *T*-test was used when measurement data obey normal distribution, and rank sum test was used when it did not obey normal distribution. *χ*^2^ test was used to compare the classified counting data. Repeated measurement data were analyzed by repeated measurement analysis of variance. Main effect test results were used when there was no interaction, and simple effect analysis was carried out when there was interaction. *P* < 0.05 indicated that the difference between groups is statistically significant.

## 3. Results

### 3.1. Comparison of Curative Effect between Two Groups

Comparing the curative effect, the curative effect of the research cohort was 93.33% (28/30), which was upregulated remarkably than that of the control group 66.67% (20/30), and the difference was statistically significant (*P* < 0.05). All results were shown in Figure 1.

### 3.2. Comparison of the Incidence of Complications

The incidence of corneal opacity, lens opacity, preretinal and vitreous hemorrhage, endophthalmitis, and traction retinal detachment in the research group was greatly lower than the control group, and the difference was statistically significant (*P* < 0.05). All results were shown in Figure 2.

### 3.3. Comparison of Intraocular Pressure at Different Time

Following treatment, the IOP of the two groups decreased at different times, and the IOP of 1 min, 10 min, and 30 min in the research group was considerably lower than that of the control. All results were shown in Table 1.

### 3.4. Comparison of Serum IL-17A Levels

After treatment, the level of serum IL-17A in both groups decreased, and the level of serum IL-17A in the research group was remarkably downregulated than control group. All results were shown in Table 2.

The article "The Effects of Combuxil and Leizumab on Retinal Function and Serum Interleukin-17A in Premature Infants with Retinopathy" was published in 2022. Journal: Comput Math Methods Med.

## 4. Discussion

Epidemiological survey results show that more than 1300 million premature infants born worldwide survived through infancy in 2010 [18]. It is estimated that more than 1.8 million premature infants suffer from varying degrees of ROP, of which more than 50000 may cause visual impairment [19–22]. The “first ROP blindness epidemic” occurred in industrialized countries in the 1940s and 1950s, mainly affecting premature infants in the United States. Unmonitored oxygen supplementation is a major risk factor for premature infants [18]. At that time, it has been carried out for 6 years since 1940 for the presence of bilateral eye-related lesions (the growth of embryonic connective tissue behind the lens, only a few retinal vessels full of blood flow, the presence of intravitreous arteries, abnormal iris color, retinal folds, and retinal detachment. The investigation of the project with different severity (only a few traces after the lens to the extent of extensive involvement) found that extremely premature infants were abnormally common. At that time, many eye signs were considered to be caused by such important and abnormal eye development, such as retinal retardation or lack, early shallowness of the anterior chamber, corneal lens adhesion, corneal opacity, and congenital glaucoma. ROP is not only the leading cause of sexual blindness in children but also one of the important eye diseases leading to white pupil sign [19, 20]. However, premature infants have no choice but to use the auxiliary oxygen therapy of inhaling high concentration oxygen. It is an important measure to save the lives of premature infants, but it is a risk factor for retinopathy of premature infants [21–23]. This study was to investigate the effects of Compaximab and raizumab on retinal function and serum interleukin-17A level in retinopathy of prematurity.

Compared with after birth, the fetus is in a state of hypoxia in the womb. When babies are born prematurely, relative oxygen levels sometimes will increase even if oxygenation is at normal environmental levels. Supplementary oxygen therapy with high supplementation of oxygen may damage capillaries and make the development of retina in an environment of high oxygen concentration, which leads to the delay of normal retinal growth and development. However, once the auxiliary system of oxygen therapy is removed, the retina of children will immediately be in a relatively anoxic concentration environment. The pathological neovascularization will grow excessively in order to balance oxygen supply and demand. Therefore, the mismatch of oxygen demand in the developing retina, coupled with preterm delivery and other factors can affect normal retinal angiogenesis, leading to the occurrence of ROP [24].

The article "The Effects of Combuxil and Leizumab on Retinal Function and Serum Interleukin-17A in Premature Infants with Retinopathy" was published in 2022. Journal: Comput Math Methods Med.

Retinal vessels first proliferate and differentiate from fusiform cells to endothelial cells in the inner layer of the retina, while the inner vessels develop into outer vessels by budding. Angiogenesis is regulated by many factors, and there are many regulatory factors that promote angiogenesis. So far, vascular endothelial growth factor (VEGF) is the strongest growth factor found to promote angiogenesis [25]. It can induce angiogenesis, increase vascular permeability, degenerate extracellular matrix, and proliferate vascular endothelial cells. At the same time, it is also the main cytokine that leads to abnormal vascular and fibrous vascular proliferation of ROP [26, 27], which can promote retinal neovascularization. In recent years, more and more studies have found the importance of development and pathogenesis of ROP [28]. Vitreous injection of anti-VEGF is also used more and more to treat ROP [29–31].

Among these anti-VEGF drugs, razumab is a specific, recombinant humanized IgG1kappa homologous monoclonal antibody fragment with molecular weight 48kD, which has a strong affinity for all subtypes of VEGF [32]. Razumab can block VEGF-A quickly and for a long time, thus reducing vascular endothelial cell proliferation and vascular permeability, inhibiting angiogenesis and repairing the blood-retinal barrier [33]. The drug has been approved for market in many countries at home and abroad and has been approved for clinical application in wet (neovascular) ARMD in China [34]. In the related ROP treatment studies, the RAINBOW study has proved the efficacies and safeties of intravitreal razumab, which makes intravitreal injection of anti-VEGF drug razumab gradually become an important means. Many studies have reported that vitreous injection of anti-VEGF razumab is generally effective [35]. Chandra treated 52 eyes with razumab, and 8 eyes (15.38%) in the razumab group needed additional retinal laser photocoagulation, anti-VEGF, external scleral ligation, or vitrectomy [36]. The study of Biju et al. included 283 eyes of 145 patients [37]. Vascular lesions disappeared in 266 eyes (94.0%) after intravitreal injection of razumab, and another 152 eyes received additional laser or surgical treatment.

Interleukin 17A (IL-17A) is a cytokine marker produced by T helper cell 17 (Th17) and a cytokine marker of the IL-17 family. There is increasing evidence that IL-17 mediates neovascularization in ophthalmopathy, but the specific mechanism is still controversial [38]. The possible role of IL-17A in neovascularization is realized through the regulatory network of cytoskeleton remodeling, VEGF-related cytokines and complement components. IL-17A may be an indirect angiogenic factor. On the one hand, its angiogenic effect involves the enhancement of cell migration and angiogenesis, which depends on the cytoskeleton remodeling mediated by PI3K-Rac1 and RhoA. On the other hand, IL-17A can increase the capillary formation of vascular endothelial cells by enhancing the migration, proliferation, and expression of VEGF, IL-6, and IL-8.

The article "The Effects of Combuxil and Leizumab on Retinal Function and Serum Interleukin-17A in Premature Infants with Retinopathy" was published in 2022. Journal: Comput Math Methods Med.

Conbercept, is a fusion protein containing extracellular domain of VEGF receptor 1 and 2 independently developed in China, which can bind to VEGF with high affinity and exert its effect. Conbercept can block all homo-types of VEGF with high binding affinity for VEGF-An and a longer half-life in the vitreous cavity [39]. It is necessary to add other differences that may exist in the treatment of ROP as mentioned in the introduction.

VEGF is a protein that can cause macular edema [20]. Many studies have shown that the expression of VEGF in vitreous cavity of patients with RVO is higher than that of normal people [21, 22]. Therefore, suppressing or reducing the expression of VEGF should be a good strategy for the treatment of ROP. Vitreous injection of anti-VEGF drugs has become the main measure for the treatment of ROP at home and abroad. The most widely used anti-VEGF drugs in China are razumab and Combuxil. Razumab has been approved for the treatment of ROP by FDA for many years since 2007 and 2010, showing its good efficacy.

With the widespread use of razumab and Compaximab, adverse reactions of razumab and Compaximab include accelerated cataract formation, thrombosis, and vitreous hemorrhage [23, 24]. The analysis shows that compared with Combuxil, razumab can attenuate neovascularization retinopathy by inhibiting the expression of IL-17A and act on RORIL-17A axis to reduce the production of VEGF by reducing the proliferation of microglia and Muller glial cells. At the same time, it can prevent the loss of ganglion cells, further regulate intraocular pressure, and improve the prognosis of patients [40]. This study still has some shortcomings. Firstly, the quality of this study is limited due to the small sample size we included in the study. Secondly, this research is a single-center study, and our findings are subject to some degree of bias. Therefore, our results may differ from those of large-scale multicenter studies from other academic institutes. This research is still clinically significant and further in-depth investigations will be carried out in the future.

To sum up, intravitreal injection of razumab is an effective treatment for retinopathy of prematurity, which can effectively improve the retinal function of infants. The level of serum interleukin-17A can be reduced and intraocular pressure can be regulated, which is safe and effective.

The article "The Effects of Combuxil and Leizumab on Retinal Function and Serum Interleukin-17A in Premature Infants with Retinopathy" was published in 2022. Journal: Comput Math Methods Med.

## Figures and Tables

**Figure 1:** The comparison of the curative effect between two groups. The blue bar is indicating the invalid cases following treatment; the orange bar is indicating the effective cases after therapy.

**Figure 2:** The comparison of the incidence of adverse reactions between two groups. The blue bar is indicating the control group; the orange bar is indicating the research group.

**Table 1:** Intraocular pressure between the two groups at different times $\left[\bar{x}\pm \text{s}\right]$.

Grouping	*N*	Before treatment	After treatment 1 min	After treatment 10 min	After treatment 30 min
Control group	30	16.59 ± 2.21	25.96 ± 3.37	18.39 ± 3.45	16.59 ± 3.31
Research group	30	16.53 ± 2.34	20.39 ± 2.21	16.49 ± 2.29	14.34 ± 1.21
*T* value		0.102	7.570	2.513	3.496
*P* value		>0.05	<0.05	<0.05	<0.05

**Table 2:** Serum IL-17A levels between the two groups [$\bar{x}\pm s$, pg/ml].

Grouping	*N*	Before treatment	After treatment 1d	After treatment 15d
Control group	30	473.95 ± 54.22	406.29 ± 16.34	379.59 ± 24.94
Research group	30	476.39 ± 50.91	363.94 ± 43.42	324.01 ± 31.56
*t* value		0.179	4.999	7.568
*P* value		>0.05	<0.05	<0.05

## Data Availability

The datasets used and analyzed during the current study are available from the corresponding author upon reasonable request.
